The article "Comparison of the Efficacy and Complications of Soft Ureteroscopy Lithotripsy and Percutaneous Nephrolithotomy in the Treatment of Urinary Calculi: A Systematic Review and Meta-analysis" was retracted in 2023. Reasons: unreliable results or conclusions; concerns about the data; concerns about the results or conclusions; concerns about the peer review.

# Comparison of the Efficacy and Complications of Soft Ureteroscopy Lithotripsy and Percutaneous Nephrolithotomy in the Treatment of Urinary Calculi: A Systematic Review and Meta-analysis

**DOI:** 10.1155/2022/5829205

**Published:** 2022-07-01

**Authors:** WenLong Han, Jing Ge, Xianlin Xu

**Affiliations:** Department of Urology, Sir Run Run Hospital, Nanjing Medical University, 211100, China

## Abstract

**Objective:**

To systematically evaluate the efficacy and complications of soft ureteroscopic lithotripsy (SUL) and percutaneous nephrolithotomy (PCNL) in the treatment of urinary calculi and to provide evidence-proof medicine basis for the popularization and application of flexible ureteroscopic lithotripsy.

**Methods:**

PubMed, EMBASE, ScienceDirect, Cochrane Library, China knowledge Network Database (CNKI), China VIP Database, Wanfang Database, and China Biomedical Literature Database (CBM) were searched for randomized controlled trials (RCT) related to soft ureteroscopic lithotripsy and percutaneous nephrolithotomy in the treatment of urinary calculi from Jan. 2010 to Mar. 2022. The bias risk of each included literature was assessed according to the standard of Cochrane manual 5.1.0. The collected data were meta-analyzed by RevMan 5.4 statistical software.

**Results:**

Ultimately, 6 RCT (a total of 794 samples) were included for meta-analysis. Heterogeneity test results of stone clearance rate were chi^2^ = 2.44, df = 5, *P* = 0.79 > 0.05, and *I*^2^ = 0%, indicating none obvious heterogeneity among the included research data. The test of WMD was *Z* = 2.11 (*P* = 0.03). It could be considered that compared with PCNL in the treatment of urinary calculi, SUL had a higher stone clearance rate in patients with urolithiasis. Secondly, heterogeneity test of operation time was chi^2^ = 184.95, df = 5, *P* < 0.00001, and *I*^2^ = 97%. The results of heterogeneity test of intraoperative blood loss displayed chi^2^ = 645.47, df = 5, *P* < 0.00001, and *I*^2^ = 99%. Then, heterogeneity test results of postoperative hospital stay existed chi^2^ = 57.37, df = 5, *P* < 0.00001, and *I*^2^ = 91% with an obvious heterogeneity. According to the results of this analysis, it could be considered that compared with PCNL in the treatment of urolithiasis, the operation time of SUL in the treatment of urolithiasis was longer, but the amount of intraoperative bleeding and postoperative hospital stay was significantly reduced. The results of heterogeneity of stress index level NE showed as chi^2^ = 0.32, df = 2, *P* = 0.85 > 0.05, and *I*^2^ = 0%, and COR was chi^2^ = 1.09, df = 1, *P* = 0.30 > 0.05, and *I*^2^ = 8%. It showed that there was no obvious heterogeneity. The heterogeneity of ACTH was chi^2^ = 390.36, df = 2, *P* < 0.00001, and *I*^2^ = 99%, suggesting obvious heterogeneity. The test of combined effect dose WMD was *Z* = 21.90, 4.50, and 15.42, (*P* < 0.00001). It could be considered that there was a statistical difference in the WMD of stress response between patients with urinary calculi treated by soft ureteroscope and percutaneous nephrolithotomy, indicating that the stress response of patients with urinary calculi treated with SUL is less than that of PCNL. For the heterogeneity test of serum creatinine level, NE showed chi^2^ = 0.78, df = 2, *P* = 0.68 > 0.05, and *I*^2^ = 0% without obvious heterogeneity, and the combined effect dose WMD is analyzed by random effect model. The test of combined effect dose WMD was *Z* = 4.22 (*P* < 0.00001). It can be considered that the improvement of serum creatinine level in patients with urolithiasis treated with SUL was better than that of PCNL. The results of heterogeneity test on the safety of operation are as follows: chi^2^ = 13.76, df = 5, *P* = 0.02, and *I*^2^ = 64%, indicating obvious heterogeneity among the included research data. The combined effect dose of WMD was *Z* = 5.53 (*P* < 0.00001). This could be considered that soft ureteroscopic lithotripsy had higher safety and less postoperative complications than percutaneous nephrolithotomy in the treatment of urinary calculi. An inverted funnel chart was used to analyze the publication bias of the study with stone clearance rate as the outcome index. The results showed that the figure was not completely symmetrical and the Egger's test showed that the figure was *P* = 0.0005 < 0.001. It was suggested that there may be a certain degree of publication bias.

**Conclusion:**

PCNL and SUL can achieve higher stone clearance rate in the treatment of renal calculi. However, SUL has the advantages of less intraoperative bleeding, short stress reaction and postoperative hospital stay, less damage to renal function, and low incidence of complications, which is beneficial to the rapid recovery of patients after operation. More studies with higher methodological quality and longer intervention time are needed to further verify.

## 1. Introduction

Renal calculus is one of the most common benign diseases in urology [1]. With the improvement of people's life quality, the change of dietary structure is not what it used to be [2]. At present, China is one of the three high incidence areas of urinary calculi in the world with an overall incidence of 1%-5%, and there are obvious regional differences. Calculi can be located in the transitional zone of renal pelvis and ureter, renal pelvis, and calyx, among which calculi in renal pelvis or calyx are the most common, while stones in renal parenchyma are rare. So far, there is still no unified conclusion on the mechanism of renal stone formation, in which supersaturated urine can promote crystal formation; lack of inhibitors and the existence of nuclear matrix are the main factors of stone formation. Untreated kidney stones often cause complete or incomplete urinary obstruction, leading to hydronephrosis and urinary tract infections and, in severe cases, even acute or chronic kidney failure. Therefore, kidney stone disease should be detected and treated as soon as possible. In the past, traditional Chinese medicine or surgical open surgery was mainly used in the treatment of kidney stones, but the effect of drugs was often uncertain. Traditional surgery requires a 20 cm incision into the kidney to remove stones, which can achieve ideal stone removal effect, but it has some disadvantages, such as large trauma and high incidence of complications.

Recently, a variety of minimally invasive treatments for renal calculi have been carried out in China. A large number of new procedures such as extracorporeal shock wave lithotripsy (ESWL), soft ureteroscopy lithotripsy (SUL), and percutaneous nephrolithotomy (PCNL) have emerged, which opened a new era in the treatment of renal calculi. ESWL is currently recognized as one of the most minimally invasive and safe methods for the treatment of renal calculi [3], but the success rate is closely related to the specific location, diameter, hardness, and anatomical structure of renal pelvis and calyx [4]. Repeated lithotripsy failure will cause kidney and surrounding tissue and organ damage and other complications. A large number of patients with kidney stones in urology clinics are concerned about the effectiveness of stone removal after ESWL and end up choosing other lithotripsy options. The consensus of experts on soft ureteroscopic lithotripsy in China in 2020 points out that SUL is recommended to treat renal calculi with diameter ≤ 2 cm and upper ureteral calculi. The consensus also points out that residual stones after percutaneous nephrolithotomy can still be treated by SUL [5]. SUL can enter the kidney through the natural passage of the human body. Small iatrogenic trauma and low incidence of postoperative complications are its unique advantages, but improper operation during operation will also cause a series of complications, such as ureteral perforation, ureteral mucosal avulsion or even rupture, urogenic sepsis, water poisoning, ureteral stone street formation, and long-term ureteral stricture.

In recent years, flexible ureteroscope and lithotripsy auxiliary equipment are also developing rapidly. With the continuous improvement of lithotripsy auxiliary equipment such as holmium laser, ureteral conveying sheath (UAS), and stone net basket, the application of flexible ureteroscope technology has been gradually expanded [6], but we should also pay attention to the important influence of renal anatomy on SUL [7]. Domestic scholar Chen Keliang et al. compared the clinical effects of PCNL and SUL in the treatment of diameter 1.5 cm~2.5 cm renal calculi [8]. The results showed that SUL could not find stones in the treatment of lower calyceal calculi, resulting in significantly long operation time, and postoperative stone clearance rate (SFR) was much lower than that of PCNL. At present, PCNL is the first choice for the treatment of large renal calculi (>2 cm) and complex and staghorn renal calculi. Especially, when complicated with renal pelvis and lower calyx stones with severe hydronephrosis, it has unique advantages compared with other stone removal methods. In the consensus of experts on percutaneous nephrolithotripsy in China in 2020, it is recommended that for lower calyx stones > 1.5 cm or calyceal stones with clinical symptoms, PCNL should be preferred if there is no contraindication [9]. Although the efficacy of PCNL in the treatment of renal calculi is accurate, it still needs to puncture and dilate the kidney to establish an operating channel. The damage to the kidney is relatively large and the intraoperative and postoperative complications are also increased accordingly. The incidence of intraoperative and postoperative bleeding and blood transfusion in patients with sex PCNL was 11.2%-17.5%, the postoperative fever rate was 21.0%-32.1%, the incidence of urinary sepsis was 0.3%-4.7%, the probability of postoperative urinary extravasation was 7.2%, and the incidence of intraoperative colonic injury and pleural injury was 0.2%-0.8% and 3.1%, respectively [10].

Both SUL and PCNL are available surgical options for the treatment of renal calculi with diameter ≤ 2 cm, but each of the two surgical methods has its own advantages and disadvantages [11]. In order to achieve better outcomes, the specific location, size, and family economic status of the stones should be comprehensively considered. In this study, we comprehensively evaluated the research articles of PCNL and SUL in the treatment of urinary calculi by meta-analysis.

## 2. Research Contents and Methods

### 2.1. Sources and Retrieval Methods of Documents

The Chinese Journal full-text Database (CNKI), VIP full-text Database (VIP), Wanfang Database, and Chinese Biomedical Literature data (CBM) were searched, and the relevant Chinese journals, conference papers, and degree papers were searched. With the method of literature review, the relevant data of SUL and PCNL patients with urinary calculi in China were collected. Literatures were conducted in the form of free words and subject words with the key words of soft ureteroscopic lithotripsy, percutaneous nephrolithotomy, and urinary calculi from Jan. 2010 to Mar. 2022.

### 2.2. Inclusion and Exclusion Criteria of Literature

#### 2.2.1. Literature Inclusion Criteria

(1) Study type: all the randomized controlled trials (RCTs) of SUL and PCNL in the treatment of urolithiasis in China. The language was limited to Chinese. (2) Participants: patients with urolithiasis were diagnosed as renal calculi by imaging examination, the stone diameter was ≤2.0 cm, and conformed to the indication of operation. (3) Intervention: SUL was used in the observation group and PCNL was used in the control group.

#### 2.2.2. Document Exclusion Criteria

(1) The research type was not RCT. (2) The data report was incomplete and the data could not be used. (3) The content of the study was repeated. (4) The evaluation of the curative effect of the study was not significant

### 2.3. Quality Evaluation and Data Extraction

#### 2.3.1. Bias Risk Assessment Included in the Study

The bias risk assessment tool recommended by Cochrane system Review Manual 5.3 was used for evaluation.

#### 2.3.2. Literature Screening and Data Extraction

Two researchers independently selected the literature, data extraction, quality evaluation, and cross-check. In case of differences, discussion or solution or asking the third researcher was performed to assist in judgment. NoteExpress documental software and Excel office software were used to manage and extract research data. If the data included in the literature was incomplete, we contacted the author of this article to supply it. The content of data extraction included (1) basic information, including author(s), publication time, and number of cases; (2) intervention measures, such as dose and course of treatment; and (3) outcome index.

### 2.4. Statistical Processing

Meta-analysis was carried out by RevMan 5.3 software. Relative risk (OR) was used as the effect index for counting data and mean difference (MD) was used as the effect index for measurement data. The point estimate and 95% confidence interval (CI) of each effect were given. *χ*^2^ test was used for heterogeneity test and *I*^2^ was used to judge the heterogeneity. If there was no heterogeneity, the fixed effect model was used. If there was heterogeneity, subgroup analysis or sensitivity analysis or descriptive analysis was used and the random effect model was used. The difference was statistically significant (*P* < 0.05).

## 3. Results and Analysis

### 3.1. The Results of Literature Retrieval and the Basic Situation of Literature Inclusion

A total of 1324 articles were obtained by searching the computer database, and 263 articles were obtained after repeated studies were excluded. Through the preliminary screening of literature titles and abstracts, a total of 76 related literatures were obtained. Irrelevant studies, reviews, case reports, and noncontrol literatures were excluded, and 48 articles were included. Then, we read the full text carefully and excluded 42 articles with incomplete data and no main outcome indicators. Finally, 6 randomized controlled trials were included [11–16]. A total of 794 samples were analyzed by meta-analysis. The basic features included in the literature are shown in Table 1.

### 3.2. Evaluation of the Quality of Methodology Included in the Literature

All the six RCT literatures included in this meta-analysis reported the baseline status of patients. One of the RCT mentions “random allocation” without any explanation. The detailed intervention measures and follow-up time were given in the 6 studies included. However, the blind method and the number and reasons of those who lost follow-up or withdrew were not described in detail. According to the Jadad scale, we found that the 6 RCTs were less than or equal to 2 points. It shows that the publication bias is low and the quality of the article is high. The risk bias analysis is shown in Figures 1 and 2.

Showing risk of bias as either low (green), unclear (yellow), or high (red) for included studies, for random sequence generation, allocation concealment, blinding of participants and personnel, blinding of outcome assessment, incomplete outcome data, selective reporting, or other bias.

### 3.3. Results of Meta-analysis

#### 3.3.1. The Stone Clearance Rate

A total of 794 samples were collected from 6 RCT studies. The results of meta-analysis of the stone clearance rate of the observation group and the control group were as follows: chi^2^ = 2.44, df = 5, *P* = 0.79 > 0.05, and *I*^2^ = 0%, indicating that there is no obvious heterogeneity between the included data; it will not affect the effectiveness of meta-analysis, so the fixed effect model is used to analyze the combined effect dose of WMD. According to the analysis of Figure 3, the test of WMD was *Z* = 2.11 (*P* = 0.03). According to the results, it could be considered that there was a statistical difference in the WMD of the stone clearance rate between SUL and PCNL. The 95% confidence horizontal line of WMD fell to the right of the invalid line, indicating that the stone clearance rate of patients with urinary calculi treated by soft ureteroscopic lithotripsy was remarkably higher than that of percutaneous nephrolithotomy (Figure 3).

#### 3.3.2. The Surgical Indexes

The results of meta-analysis of the operation conditions of the observation group and the control group were as follows: (1) heterogeneity test of operation time was chi^2^ = 184.95, df = 5, *P* < 0.00001, and *I*^2^ = 97%; (2) heterogeneity test of intraoperative blood loss was chi^2^ = 645.47, df = 5, *P* < 0.00001, and *I*^2^ = 99%; (3) heterogeneity test of length of stay in hospital was chi^2^ = 57.37, df = 5, *P* < 0.00001, and *I*^2^ = 91%. Great heterogeneity was found among the included research data, indicating that there is obvious heterogeneity between the included research data; the explanation will affect the effectiveness of meta-analysis, so the random effect model is used to analyze. According to Figures 4–6, the test of combined effect dose WMD was *Z* = 32.25, 62.82, and 26.80 (*P* < 0.00001). It could be considered that there were significant differences in operation time, intraoperative blood loss, and hospital stay between SUL and PCNL, which indicated that the operation time of SUL in the treatment of urolithiasis was greatly longer than that of PCNL, but the intraoperative blood loss and postoperative hospital stay were remarkably reduced (Figures 4–6).

#### 3.3.3. The Stress Index Level

Meta-analysis results of stress index level between observation group and control group are as follows: heterogeneity test results: NE: chi^2^ = 0.32, df = 2, *P* = 0.85 > 0.05, and *I*^2^ = 0% and COR: chi^2^ = 1.09, df = 1, *P* = 0.30 > 0.05, and *I*^2^ = 8%. It showed that there was no obvious heterogeneity among the included research data. ACTH is as follows: chi^2^ = 390.36, df = 2, *P* < 0.00001, and *I*^2^ = 99%. It displayed that there was obvious heterogeneity in the included research data, indicating that there is obvious heterogeneity between the included research data; the explanation will affect the effectiveness of meta-analysis, so the combined effect dose WMD was analyzed by random effect model. According to the analysis of Figures 7–9, the test of combined effect dose WMD was *Z* = 21.90, 4.50, and 15.42 (*P* < 0.00001). According to this analysis, it could be considered that there was a statistical difference in the WMD of stress response between SUL and PCNL, indicating that the stress response of patients with urolithiasis treated with SUL was less than PCNL (Figures 7–9).

#### 3.3.4. Serum Creatinine Level

The heterogeneity test results were as follows: NE: chi^2^ = 0.78, df = 2, *P* = 0.68 > 0.05, and *I*^2^ = 0%. It showed that there is no obvious heterogeneity between the included data; it will not affect the effectiveness of meta-analysis, so the fixed effect model is used to analyze the combined effect dose of WMD. According to Figure 10, the test of combined effect dose WMD was *Z* = 4.22 (*P* < 0.00001). It could be considered that there was a significant difference in the level of serum creatinine between SUL and PCNL, indicating that the improvement of serum creatinine in patients with urolithiasis treated with SUL was better than that of PCNL (Figure 10).

#### 3.3.5. Postoperative Complications

The postoperative complications reported in the 6 articles included in this study included postoperative infection, bleeding, high fever, urinary tract injury, and renal colic. Meta-analysis of surgical safety was conducted between the observation group and the control group. The results of heterogeneity test were as follows: chi^2^ = 13.76, df = 5, *P* = 0.02, and *I*^2^ = 64%, showing that there was significant heterogeneity among the included research data, indicating that there is obvious heterogeneity between the included research data; the explanation will affect the effectiveness of meta-analysis, so the combined effect dose WMD was analyzed by random effect model. According to Figure 11, the test of combined effect dose WMD was *Z* = 5.53 (*P* < 0.00001). According to the results, it could be considered that compared with percutaneous nephrolithotomy in the treatment of patients with urinary calculi, soft ureteroscopic lithotripsy had higher safety and fewer postoperative complications (Figure 11).

#### 3.3.6. Publication Bias Analysis

The inverted funnel chart was used to analyze the publication bias of the study with stone clearance rate as the outcome index (Figure 12). The results showed that the figure was not completely symmetrical between left and right. Egger's test shows *P* = 0.0005 < 0.001, suggesting that there may be a certain degree of publication bias.

## 4. Analysis and Discussion

Urolithiasis is one of the most common diseases in urology with a global incidence of about 5% to 15% [17]. Kidney stone is a common clinical disease of urinary calculi, but complex kidney stone is more difficult in the process of surgical treatment. Minimally invasive surgery has a history of more than 30 years in the treatment of renal calculi. Before minimally invasive surgery was widely used, there were two main methods for the treatment of renal calculi [18]. The function of the kidney is seriously damaged. There are more intraoperative and postoperative complications, and the effect of drug therapy on stone dissolution is even more disappointing to clinicians. Therefore, the two traditional treatments are gradually replaced with the development of minimally invasive surgery. Minimally invasive surgery is widely respected by clinicians because of its advantages such as short operation time, less trauma, less complications, and quick recovery after operation. At present, the minimally invasive surgical techniques widely used for the treatment of complex renal calculi include SUL, ESWL, and PCNL. Among the above surgical techniques, SUL is compared by clinical experts as “entering through the door.” At the same time, it can safely enter the renal pelvis (living room) and calyx (holiday) of the kidney, reflecting the advantages of soft lens technology [19, 20]. It is closer to being “noninvasive,” making it an important part of the minimally invasive surgical treatment of upper urinary tract stones and even of complex kidney stones. Fifty years have passed since Marshall first used flexible scopes to examine ureteral stones in 1946. In the last two decades, the application of flexible microscopy techniques in the management of complex kidney stones has received increasing attention from clinicians.

Subsequently, the soft ureteroscope is widely used in clinical examination and surgical treatment. Soft lens can be divided into two types [21], one is only for examination, and the other can be used not only for examination but also for the treatment of stones and other related diseases. The soft microscope device used for examination only looks like a catheter with a thin core and no manipulable channels. This flexible mirror is used for observation only during examination and cannot be treated. This kind of soft mirror is rarely used at present. Now, the most widely used is the flexible ureteroscope with treatment pathway, which has different types of external diameter from 9.3F to 2.3F.

Compared with ESWL and PCNL, SUL has the advantages of less trauma, faster recovery, and lower complications in the treatment of upper urinary tract calculi < 2 cm [22]. In clinical work, we should understand and master the indications and contraindications of flexible ureteroscope in order to achieve better therapeutic effect. According to the guidelines for diagnosis and treatment of Chinese Urology and Andrology Diseases (2019 Edition) [23], the indications of SUL included (1) renal calculi within 2 cm and cannot be seen on X-ray or cannot be located by ESWL, (2) patients with pathological obesity, (3) severe spinal deformities and unable to establish effective PCNL working channels, (4) hard stones, (5) incarcerated lower calyx stones, (6) calculi in the diverticulum, and (7) stones in the lower calyx after ESWL treatment. The contraindications included (1) patients with systemic hemorrhagic diseases that cannot be effectively controlled due to severe abnormal blood coagulation; (2) patients with severe cardiopulmonary insufficiency before operation; (3) patients with high risk of operation and anesthesia; (4) patients with severe urinary tract infection indicated by urine routine or urine culture; (5) patients with severe urethral stricture, deformity, and tumor leading to endoscopic failure; and (6) patients with severe hip deformities, which lead to difficulties in surgical posture.

At present, scholars at home and abroad generally believe that for upper urinary tract stones with diameter > 2 cm or even staghorn calculi, PCNL has more advantages than SUL in one-time stone removal rate [24, 25]. Generally speaking, the larger the diameter of the stone, the greater the damage to the kidney and directly affect the effect of intraoperative lithotripsy and postoperative stone clearance. Sari et al. conducted a meta-analysis of the clinical data of 455 patients with renal calculi treated with SUL > 2 cm [26]. The results showed that when the diameter was in the range of 2~3 cm, the postoperative stone clearance rate was 95.7%. When the stone diameter > 3 cm, the postoperative stone removal rate can reach 84.6%. This result has provided an objective and real theoretical basis for SUL in the treatment of upper urinary tract stones > 2 cm. Therefore, when SUL is used to treat upper urinary tract calculi in clinical work, especially when the diameter of renal calculi is more than 3 cm, PCNL should be given priority if there is no obvious taboo, so as to avoid affecting the effect of postoperative stone clearance due to excessive stone diameter. Yi and Yun suggested that 80 patients with kidney stones with diameter> 2 cm were treated through SUL, the stone clearance rate could reach 75%, and the total postoperative clearance rate could be as high as 91.7% [27]. There were also no serious complications after operation, which was consistent with foreign literature reports. For upper urinary tract calculi with diameter ≤ 2 cm, SUL and PCNL have the same effect on stone clearance rate [28, 29]. However, the two surgical methods have their own advantages and disadvantages, and reasonable choices should be made according to the actual situation in clinical work. If there are contraindications to PCNL, we can consider changing to SUL treatment. There is still a high postoperative stone clearance rate, and it is also a safe and effective clinical treatment option [30].

Ultimately, 6 RCT (a total of 794 samples) were included for meta-analysis in our analysis. Heterogeneity test results of stone clearance rate were chi^2^ = 2.44, df = 5, *P* = 0.79 > 0.05, and *I*^2^ = 0%, indicating none obvious heterogeneity among the included research data. The test of WMD was *Z* = 2.11 (*P* = 0.03). It could be considered that compared with PCNL in the treatment of urinary calculi, SUL had a higher stone clearance rate in patients with urolithiasis. Secondly, heterogeneity test of operation time was chi^2^ = 184.95, df = 5, *P* < 0.00001, and *I*^2^ = 97%. The results of heterogeneity test of intraoperative blood loss displayed chi^2^ = 645.47, df = 5, *P* < 0.00001, and *I*^2^ = 99%. Then, heterogeneity test results of postoperative hospital stay existed chi^2^ = 57.37, df = 5, *P* < 0.00001, and *I*^2^ = 91% with an obvious heterogeneity. According to the results of this analysis, it could be considered that compared with PCNL in the treatment of urolithiasis, the operation time of SUL in the treatment of urolithiasis was longer, but the amount of intraoperative bleeding and postoperative hospital stay were significantly reduced. The results of heterogeneity of stress index level NE showed as chi^2^ = 0.32, df = 2, *P* = 0.85 > 0.05, and *I*^2^ = 0%, and COR was chi^2^ = 1.09, df = 1, *P* = 0.30 > 0.05, and *I*^2^ = 8%. It showed that there was no obvious heterogeneity. The heterogeneity of ACTH was chi^2^ = 390.36, df = 2, *P* < 0.00001, and *I*^2^ = 99%, suggesting obvious heterogeneity. The test of combined effect dose WMD was *Z* = 21.90, 4.50, and 15.42 (*P* < 0.00001). It could be considered that there was a statistical difference in the WMD of stress response between patients with urinary calculi treated by soft ureteroscope and percutaneous nephrolithotomy, indicating that the stress response of patients with urinary calculi treated with SUL is less than that of PCNL. Heterogeneity test of serum creatinine level is as follows: NE showed chi^2^ = 0.78, df = 2, *P* = 0.68 > 0.05, and *I*^2^ = 0% without obvious heterogeneity and the combined effect dose WMD is analyzed by random effect model. The test of combined effect dose WMD was *Z* = 4.22 (*P* < 0.00001). It can be considered that the improvement of serum creatinine level in patients with urolithiasis treated with SUL was better than that of PCNL. The results of heterogeneity test on the safety of operation are as follows: chi^2^ = 13.76, df = 5, *P* = 0.02, and *I*^2^ = 64%, indicating obvious heterogeneity among the included research data. The combined effect dose of WMD was *Z* = 5.53 (*P* < 0.00001). This could be considered that soft ureteroscopic lithotripsy had higher safety and less postoperative complications than percutaneous nephrolithotomy in the treatment of urinary calculi. An inverted funnel chart was used to analyze the publication bias of the study with stone clearance rate as the outcome index. The results showed that the figure was not completely symmetrical and the Egger's test showed that the figure was *P* = 0.0005 < 0.001. It was suggested that there may be a certain degree of publication bias.

## 5. Conclusion

To sum up, for the treatment of patients with urinary calculi, SUL has the advantages of more minimally invasive, less complications, less postoperative hospital stays, and rapid recovery. However, the selection of surgical methods needs to the plans of corresponding treatment according to the specific conditions of the patients. The growing of studies with higher methodological quality and longer intervention time are still needed to further verify.

## Figures and Tables

**Figure 1:** Summary of risk of bias. Showing risk of bias as either low (green), unclear (yellow), or high (red) for included studies.

**Figure 2:** Risk of bias assessment of included studies.

**Figure 3:** Forest plot of meta-analysis of stone clearance rate.

**Figure 4:** Forest plot of meta-analysis of operation time.

**Figure 5:** Forest plot of meta-analysis of amount of intraoperative bleeding.

**Figure 6:** Forest plot of meta-analysis of length of hospital stay.

**Figure 7:** Forest plot of meta-analysis of NE level.

**Figure 8:** Forest plot of meta-analysis of ACTH level.

**Figure 9:** Forest plot of meta-analysis of COR level.

**Figure 10:** Forest plot of meta-analysis of serum creatinine level.

**Figure 11:** Forest plot of meta-analysis of postoperative complications.

**Figure 12:** Inverted funnel chart of stone clearance rate after ureteroscopy lithotripsy.

**Table 1:** Basic characteristics of literature.

Include the literature	Year of publication	N (C/T)	Intervention method		Outcome index	Experimental time	Whether it is random or not	Whether it is blind or not
			C	T				
Liu Gang	2022	26/26	Percutaneous nephrolithotripsy	Soft ureteroscopic lithotripsy	①②③④	3 months	Yes	No
Chen ran	2021	46/46	Percutaneous nephrolithotripsy	Soft ureteroscopic lithotripsy	①②③④⑤	3 months	Yes	No
Guo Shugang	2021	45/45	Percutaneous nephrolithotripsy	Soft ureteroscopic lithotripsy	①②④	1 month	Yes	No
Ren Chang	2018	178/152	Percutaneous nephrolithotripsy	Soft ureteroscopic lithotripsy	①②③④	4 weeks	No	No
Zhou Zhenwen	2021	40/40	Percutaneous nephrolithotripsy	Soft ureteroscopic lithotripsy	①②③④⑤	3 months	Yes	No
Song Mingze	2021	64/86	Percutaneous nephrolithotripsy	Soft ureteroscopic lithotripsy	①②④	3 months	Yes	No

①: operative index, ②: postoperative complications, ③: stress index level, ④: stone clearance rate, and ⑤: serum creatinine level.

## Data Availability

No data were used to support this study.
